RETRACTED

# Effect of Uterine Artery Ligation and Uterine Artery Embolization on Postpartum Hemorrhage Due to Uterine Asthenia after Cesarean Section and Its Effect on Blood Flow and Function of Uterine and Ovarian Arteries

**DOI:** 10.1155/2022/1337234

**Published:** 2022-03-21

**Authors:** Wufen Liu, Wei Yin

**Affiliations:** Obstetrics and Reproductive Center, Affiliated Hospital of Yunnan University, Kunming 650021, China

## Abstract

**Objective:**

To investigate the efficacy of uterine artery ligation (UAL) and uterine artery embolization (UAE) in the treatment of uterine asthenia postpartum hemorrhage (PPH) after cesarean section and its effect on uterine and ovarian artery blood flow and function.

**Methods:**

100 patients with uterine asthenia PPH after cesarean section in our hospital from January 2018 to November 2020 were randomly divided into 50 cases in the UAL group and 50 cases in the UAE group. They were followed up for 12 months. The bleeding volume, operation time, immediate hemostasis rate, and hemostasis effective rate; lochia clearance time and menstrual rehydration time; RI and S/D; and serum FSH, E2, and LH levels were compared between the two groups.

**Results:**

Compared with the UAL group, the amount of bleeding in the UAE group was significantly increased and the operation time was significantly shortened (*p* < 0.05). There was no significant difference in the immediate hemostatic rate and hemostatic effective rate between the two groups (*p* > 0.05). There was no significant difference in lochia clearance time and menstrual rehydration time between the two groups (*p* > 0.05). There was no significant difference in RI and S/D between the two groups (*p* > 0.05). Compared with before the operation, the levels of FSH and LH in the two groups decreased significantly, and the level of E2 increased significantly (*p* < 0.05). There was no significant difference between the two groups (*p* > 0.05).

**Conclusion:**

The efficacy of UAL and UAE in the treatment of PPH with uterine asthenia after cesarean section and its effect on the blood flow and function of uterine and ovarian arteries are equivalent, but the amount of bleeding in UAL is less and the operation time of UAE is shorter. The appropriate operation method can be selected according to the actual situation.

## 1. Introduction

Within 24 h of delivery of a fetus, when a hemorrhage of more than 500 mL or a cesarean section of more than 1000 mL occurs, it is called PPH. Clinical manifestations are mainly hypotension, vaginal bleeding, and other symptoms, which can cause severe anemia and hemorrhagic shock in severe cases and are one of the important causes of maternal death [1, 2]. PPH can be caused by coagulation dysfunction, rupture of the soft birth canal, placental factors, and uterine contraction weakness, among which uterine contraction weakness is the most common [3]. Cesarean section is an effective measure to rescue puerpera, fetal life and solve dystocia, and the risk of postoperative PPH is significantly higher than that of vaginal delivery [4]. At present, PPH patients are mainly treated by drugs and surgery, and for those whose hemostatic effect is not obvious, surgery is used for treatment [5]. As an effective and rapid treatment for PPH, hysterectomy is suitable for all kinds of PPH that have failed to be rescued. However, it can lead to the loss of fertility of patients and seriously damage the physical and mental health of patients. Therefore, in the treatment of PPH, more and more attention has been paid to the preservation of the uterus [6]. UAL and UAE are based on vascular treatments, which block the blood supply of the uterine artery through ligation or embolization and thus have a hemostatic effect. Both can effectively treat PPT, but both have limitations [7, 8]. At present, there are few studies on which is better than UAL or UAE in the treatment of PPH after cesarean section, which is worthy of further study. Therefore, the purpose of this study is to explore the efficacy of UAL and UAE in the treatment of postcesarean delivery PPH with uterine contraction weakness and its influence on the blood flow and function of uterine and ovarian arteries in order to provide some reference for improving the quality of life of patients with postcesarean delivery PPH with uterine contraction weakness.

RETRACTED

## 2. Data and Methods

### 2.1. General Information

A total of 100 patients with PPH after cesarean section in our hospital from January 2018 to November 2020 were selected as the study subjects, and they were divided into the UAL group (*n* = 50) and the UAE group (*N* = 50) according to the random number table method. This study was approved by the hospital's ethics committee.

### 2.2. Inclusion and Exclusion Criteria

The inclusion criteria were as follows: (1) after examination, the blood loss of all patients was 1000 mL within 24 h after fetal delivery; (2) patients who did not respond to drug treatment; (3) patients with stable vital signs; (4) patients with normal heart, liver, and kidney function; and (5) informed consent was signed by patients or their families.

The exclusion criteria were as follows: (1) patients with contraindications to UAL or UAE or who could not tolerate surgery; (2) PPH patients caused by coagulation dysfunction, soft birth canal laceration, placental factors, and other factors were excluded; (3) combined with premature ovarian failure, ovarian function decline, polycystic ovary syndrome, and other patients; and (5) patients with scar uterus.

RETRACTED

### 2.3. Methods

In the UAL group, the uterus was pulled out to the abdominal cavity by a cesarean section incision, and the uterus was pulled to one side, so that the artery was completely exposed. At the same time, the round ligament was avoided, the surgeon placed the left hand on the posterior wall of the lower uterine segment, and the round needle was passed through the outermost vascularless area of the arteriovenous plexus of the patient's uterine margin by 2∼3 cm. The distal end of the uterine artery was carefully observed with local compressions. If the distal end pulsated, the uterine artery on the contralateral side was also treated with UAL.

UAE group: patients were subjected to local anesthesia under digital subtraction angiography (GE, Innova IGS 530) until the puncture was successful. The 5 F arterial sheath (Termao, Japan) was inserted into the femoral artery, and the left uterine artery was angiographed by a 5 F Cobra catheter (Cook, USA) to ensure no extravasation of contrast media. Then, sodium chloride (H51021158), gentamicin (H42021503), and contrast agent (Chenxin Pharmaceutical Co., Ltd., H42021503) were injected into the uterine artery under fluoroscopy. Chinese medicine (approval H20063128), gelatin sponge particles (Hangzhou Ailekon Pharmaceutical Technology Co., Ltd.) of the mixture, in the embolization at the same time, pay attention to the mixture of reflux, the contralateral artery using the same method for embolization.

Patients in both groups were followed up for 12 months.

### 2.4. Observation Indicators

The observation indicators are as follows: (1) Operating-related indicators: the amount of blood loss (calculated by weighing method, visual method, and volume method), operation time, immediate hemostasis rate (bleeding stopped within 30 min after surgery), and hemostatic efficiency (no bleeding within 48 h after surgery and stable condition) were observed and compared between the two groups. (2) Postoperative recovery index: the time of lochia excretion and the time of menstrual revulsion were compared between the two groups. (3) Uterine and ovarian arterial blood flow: color Doppler ultrasonography (Mindray DC-25) was used to evaluate the vascular resistance index of the left and right uterine arteries of the 2 groups at 3–7 days after menstruation and 12 months after operation (RI, peak systolic velocity/peak diastolic velocity, and S/D). (4) Ovarian function: 3 ml of venous blood was extracted from the patients on the 2nd to 3rd day after the first menstruation before surgery and placed in the EP tube. The enzyme-linked immunosorbent assay was adopted to detect serum follicle stimulating hormone (FSH), estradiol (E2), and luteinizing hormone (LH) levels. All the kits were provided by Shanghai Fusheng Industrial Co., Ltd.

RETRACTED

### 2.5. Statistical Methods

SPSS 18.0 was used for statistical analysis. The measurement data were expressed as the mean ± standard deviation (±*S*) and tested by *T*. The enumeration data were expressed by example (*n*) or percentage (%) and tested by *χ*^2^. *p* < 0.05 indicated statistically significant difference.

## 3. Results

### 3.1. Comparison of General Data between the Two Groups

There was no statistically significant difference between the two groups in age, gestation time, gestation number, newborn weight, and maternal type (*p* > 0.05), indicating comparability, as shown in Table 1.

### 3.2. Comparison of Surgical Indicators between the Two Groups

The amount of blood loss in the UAL group was significantly less than that in the UAE group, and the operation time was significantly longer than that in the UAE group, with statistical significance (*p* < 0.05). There was no significant difference in immediate hemostasis rate and hemostasis efficiency between the two groups (*p* > 0.05), as shown in Table 2.

### 3.3. Comparison of Postoperative Recovery Indicators between the Two Groups

There was no significant difference in the net time of lochia excretion and the time of menstrual revulsion between the two groups (*p* > 0.05), as shown in Table 3.

### 3.4. Comparison of Uterine and Ovarian Arterial Blood Flow Indexes between the Two Groups

There were no significant differences in RI and S/D between the two groups (*p* > 0.05), as shown in Table 4.

### 3.5. Comparison of Ovarian Function Indexes between the Two Groups before and after Surgery

Before the operation, there were no significant differences in FSH, E2, and LH levels between the two groups (*p* > 0.05). After surgery, the levels of FSH and LH in the two groups were significantly decreased, while the level of E2 was significantly increased, with statistical significance (*p* < 0.05). There was no significant difference between the two groups (*p* > 0.05), as shown in Table 5 and Figure 1.

## 4. Discussion

PPH is a common complication after cesarean section, and uterine weakness is one of the main causes of PPH [9]. PPH is urgent and develops rapidly, requiring active and effective treatment; otherwise it may cause functional ischemia of multiple organs, hypovolemic shock, etc., and seriously affect the maternal quality of life [10]. Conservative treatment and surgical treatment are currently the main means of clinical management of PPH, and surgical treatment is performed if conservative treatment fails [11]. UAL is the most commonly used surgical method in the clinical treatment of PPH, although it has good blood control effects. However, it may block the blood supply of the uterine body, and then block the blood supply of the corresponding ovarian branches, which can cause serious damage to ovarian function and is limited in clinical application [12]. UAE is when a catheter is inserted into the femoral artery, deep into the uterine artery, and a stent, or gelatin sponge, is inserted into the artery. At the same time, it causes little trauma and can effectively preserve the body's fertility and uterus, but there are many contraindications [13]. Both UAL and UAE have certain limitations. At present, few studies have explored the efficacy of UAL and UAE in the treatment of hysteroconstrictive PPH after cesarean section and their effects on uterine and ovarian artery blood flow and function.

RETRACTED

Eggel et al. [14] showed that the effective rate in UAE treatment of PPH reached 93.50%, and the menstrual cycle recovery time was 5.6 months. Sanket and Herendael [15] showed that uterine artery ligation can effectively reduce intraoperative blood loss. In this study, the immediate hemostatic rate and hemostatic effective rate of the two groups reached more than 90%, and the time of lochia excretion and menstrual revulsion was similar in the two groups, which was basically consistent with the results of Eggel and Sanket studies, indicating that UAL and UAE have significant efficacy in the treatment of hysterostatic PPH after cesarean section. UAL can block most of the uterine blood supply, cause ischemic stimulation, promote smooth muscle contraction, and finally achieve hemostatic effect [16]. UAE is a minimally invasive surgery, which can determine the site and scope of bleeding through angiography, and perform embolization on the proximal and distal sides of the bleeding artery to timely block uterine blood supply and have an immediate hemostatic effect [17]. In addition, this study found more blood loss in the UAE group than in the UAL group. However, the operation time is shortened, and the possible reasons are analyzed: compared with UAL, UAE is simpler, but the implementation of UAE often requires the cooperation of interventional departments, thus prolonging the preoperative preparation time and resulting in increased blood loss of patients. Therefore, it is suggested that the preparation time before UAE should be shortened as much as possible [18].

RI and S/D are common hemodynamic indexes in clinical practice. RI reflects the characteristic quantity of vascular resistance. The greater the value is, the greater the vascular resistance and the more serious the blood circulation disorder. S/D is generally maintained at a dynamic equilibrium, and abnormal changes can be caused once abnormal blood flow occurs [19]. Garg [20] showed that laparoscopic uterine vascularization can maintain the stability of patients' blood flow. In this study, RI and S/D of the left and right uterine arteries in the two groups showed no significant difference. Combined with the results of Menderes' study, it was found that neither UAL nor UAE had a significant impact on the uterine and ovarian artery blood flow in patients with PPH after cesarean section. After UAL, the uterine blood supply can return to normal due to the establishment of collateral circulation. In addition, intraoperative sutures can be absorbed and have a certain tension at a certain time, which has a hemostatic effect. With proteolytic hydrolysis and uterine involution and shrinkage, sutures are gradually hydrolyzed, and the uterine artery and other blood vessels ligated will recalculate, thus having no significant influence on blood circulation [21]. After UAE, blood perfusion can be restored from the communication branch to the ovarian branch of the uterine artery. At the same time, the embolization material is absorbable gelatin sponge particles, which can reach the peripheral artery and keep the blood supply of pelvic organ collateral, so as not to affect the blood supply of uterus and ovary [22].

RETRACTED

The ovary is located in the female pelvic cavity, and its main function is to discharge and produce egg cells and secrete sex hormones so as to effectively promote and maintain the development of female characteristics. Therefore, sex hormones can effectively reflect the ovarian function of the body. FSH, E2, and LH are common sex hormones in clinical practice, and FSH plays a role in promoting follicular development and maturation. At the same time, it can cooperate with LH to induce mature follicles to secrete estrogen and ovulation, which play a role in promoting the formation of normal menstruation. FSH can be up-regulated in patients with ovarian hypoplasia, primary amenorrhea, hyporeproductive function, and so on. E2 is the most abundant and most active steroid hormone, mainly secreted from ovarian follicular granulosa cells. Once menopause, amenorrhea, ovariectomy, and ovarian dysfunction occur, the E2 level will be reduced. LH can secrete estrogen and progesterone and promote luteogenesis, and an abnormal increase of LH level may occur when menopause, oophorectomy, and premature ovarian failure occur [23]. In this study, the levels of FSH and LH decreased and E2 increased in both groups after the operation, but there was no significant difference between the two groups, indicating that UAL and UAE can promote the recovery of ovarian function in patients with PPH after cesarean section. UAL, by ligation of the uterine arcuate artery with absorbable suture, not only has an obvious hemostasis effect, but also has simple operation and little trauma, which will not have a significant impact on the uterus and promote uterine rejuvenation and functional recovery [24]. UAE can clearly observe the uterine artery variation through angiography, which provides a good display of the uterine blood supply network. At the same time, hyperselective embolization of blood supply through a microcatheter or catheter can preserve the integrity of the uterus and normal physiological function [8].

RETRACTED

## 5. Conclusion

In conclusion, both UAL and UAE can effectively treat PPH with uterine contraction after cesarean section and have a significant hemostatic effect. Both have similar effects on uterine and ovarian arterial blood flow and can effectively improve ovarian function. However, with less blood loss and a short UAE operation time, appropriate surgical procedures can be selected according to the specific situation of patients.

## Figures and Tables

**Figure 1:** Comparison of ovarian function indexes between the two groups before and after operation.

**Table 1:** Comparison of general information of the two groups of patients.

The general information	Group UAL (*n* = 50)	Group UAE (*n* = 50)	*T*	*p*
Average age (years)	29.49 ± 4.40	28.83 ± 4.73	0.372	0.708
Average gestation time (weeks)	35.56 ± 8.09	35.13 ± 8.82	0.459	0.639
Average number of pregnancies	2.62 ± 0.73	2.70 ± 0.92	1.116	0.125
Average newborn weight (kg)	3.86 ± 0.86	3.96 ± 0.97	0.854	0.397
Type of puerpera (*n* (%))	Unipara	36 (72.00)	35 (70.00)	0.454
	Multipara	14 (28.00)	15 (30.00)	0.501

**Table 2:** Comparison of operation related indexes between the two groups.

Indicators	Group UAL (*n* = 50)	Group UAE (*n* = 50)	*t*	*p*
Blood loss (mL)	1627.63 ± 403.62	1778.49 ± 429.16	5.182	0.039
Operation time (min)	60.46 ± 13.70	44.49 ± 7.43	5.867	0.032
Immediate hemostasis rate (*N* (%))	46 (92.00)	47 (94.00)	0.838	0.405
Effective rate of hemostasis (*N* (%))	48 (96.00)	49 (98.00)	0.383	0.721

**Table 3:** Comparison of postoperative recovery indexes between the two groups.

Indicators	Group UAL (*n* = 50)	Group UAE (*n* = 50)	*t*	*p*

Lochia removal time (D)	31.68 ± 2.54	31.83 ± 2.20	0.029	0.972
Period of menstruation (weeks)	41.31 ± 7.10	42.40 ± 6.73	0.245	0.784

**Table 4:** Comparison of blood flow indexes of uterine and ovarian arteries between the two groups ($\bar{x}\pm s$).

Indicators		Group UAL (*n* = 50)	Group UAE(*n* = 50)	*t*	*p*

Left uterine artery	RI	0.81 ± 0.01	0.83 ± 0.02	1.861	0.081
	S/D	12.30 ± 3.06	12.50 ± 2.82	1.525	0.116

Right uterine artery	RI	0.82 ± 0.02	0.80 ± 0.02	0.949	0.203
	S/D	12.89 ± 2.13	12.63 ± 2.86	1.316	0.354

RETRACTED

**Table 5:** Comparison of ovarian function indexes between the two groups before and after operation ($\bar{x}\pm s$).

Project		Group UAL (*n* = 50)	Group UAE (*n* = 50)

FSH (IU/L)	Before the operation	5.10 ± 1.20	5.13 ± 1.26
	After the operation	3.25 ± 0.51^*∗*^	3.16 ± 0.62^*∗*^

E2 (pmol/L)	Before the operation	18.57 ± 1.11	17.86 ± 1.10
	After the operation	33.25 ± 2.13^*∗*^	32.87 ± 2.18^*∗*^

LH (IU/L)	Before the operation	4.48 ± 0.84	4.68 ± 0.78
	After the operation	2.40 ± 0.56^*∗*^	2.23 ± 0.51^*∗*^

*Note.* Compared with that before the operation, ^*∗*^*p* < 0.05.

## Data Availability

The data used to support the findings of this study are available from the corresponding author upon request.
